# A Performance Comparison of Unsupervised Techniques for Event Detection from Oscar Tweets

**DOI:** 10.1155/2022/5980043

**Published:** 2022-05-24

**Authors:** Muzamil Malik, Waqar Aslam, Zahid Aslam, Abdullah Alharbi, Bader Alouffi, Hafiz Tayyab Rauf

**Affiliations:** ^1^Department of Computer Science & Information Technology, Islamia University of Bahawalpur, Bahawalpur, Pakistan; ^2^Department of Information Technology, College of Computers and Information Technology, Taif University, P.O. Box 11099, Taif 21944, Saudi Arabia; ^3^Department of Computer Science, College of Computers and Information Technology, Taif University, P.O. Box 11099, Taif 21944, Saudi Arabia; ^4^Centre for Smart Systems, AI and Cybersecurity, Staffordshire University, Stoke-on-Trent, UK

## Abstract

People's lives are influenced by social media. It is an essential source for sharing news, awareness, detecting events, people's interests, etc. Social media covers a wide range of topics and events to be discussed. Extensive work has been published to capture the interesting events and insights from datasets. Many techniques are presented to detect events from social media networks like Twitter. In text mining, most of the work is done on a specific dataset, and there is the need to present some new datasets to analyse the performance and generic nature of Topic Detection and Tracking methods. Therefore, this paper publishes a dataset of real-life event, the Oscars 2018, gathered from Twitter and makes a comparison of soft frequent pattern mining (SFPM), singular value decomposition and k-means (K-SVD), feature-pivot (Feat-p), document-pivot (Doc-p), and latent Dirichlet allocation (LDA). The dataset contains 2,160,738 tweets collected using some seed words. Only English tweets are considered. All of the methods applied in this paper are unsupervised. This area needs to be explored on different datasets. The Oscars 2018 is evaluated using keyword precision (*K*-Prec), keyword recall (*K*-Rec), and topic recall (*T*-Rec) for detecting events of greater interest. The highest *K*-Prec, *K*-Rec, and *T*-Rec were achieved by SFPM, but they started to decrease as the number of clusters increased. The lowest performance was achieved by Feat-p in terms of all three metrics. Experiments on the Oscars 2018 dataset demonstrated that all the methods are generic in nature and produce meaningful clusters.

## 1. Introduction

In recent years, social media networks like Twitter have become a primary source of information for reporting events that occur in real world. News posted on Twitter reaches even before the news media channels because of the localness of the users that are present at the place where the event occurs [1]. The information generated by these social networks is useful in many applications like decision making, advertisement of products, law enforcement, crisis management, predicting election results, etc. Companies also use Twitter to analyse customer interests, answer customer queries, and enhance their decision-making capabilities for business analytics. The real-time nature of the data generated by these social networks ensures fast and timely spread of information. Twitter is considered one of the main channels for expressing opinions, thoughts, interests, and sharing news and information about events and incidents due to its characteristic of being limited in size to 280 characters [2]. The average number of monthly active users around the world on Twitter is 335 million. Users post tweets in several domains such as daily routine activities, life events, local and global news, tweets about the success of their favourite celebrities, death, and winning of awards [3].

An event in the realm of social networks is considered something of interest that happens in the real world at a particular time, and users begin discussing relevant topics. The occurrence of an event causes a significant variation in the amount of text data at a particular time, which is determined by the location and individuals of the event [4]. There are several examples of events recorded by social network users in the real world such as natural disasters, formation of opinions on different political issues, sports, traffic events, and epidemic diseases [5, 6]. Thus, social network data mining became paramount to understand and anticipate the evolution of the online world. Finding topics of interest or detecting events from Twitter is a challenging task because of its high-dimensional data and conciseness where not enough information is provided. About 40% of the tweets are not related to events. For the extraction of useful details from continuous data streams, these events need to be monitored and detected.

Several techniques have been used for the detection of events that mainly fall into three categories: probabilistic models Latent Dirichlet Allocation (LDA), feature-pivot (Feat-p), and document-pivot (Doc-p) methods. The first category works on word occurrences with a probabilistic theory and calculates the topical similarity between the words; the second category clusters the documents by finding the semantic distance between documents for event detection tasks and later uses words to document distribution for clustering them together. A new way to group the documents that match the query words is to check for relevant information on Twitter using keywords, but there is no guarantee that the documents retrieved reflect the same events and often vary from user to user. However, emerging words will not yield all of the topics needed to explain the event [7]. Standard clustering-based methods are based on frequency burstiness; as these approaches are small-scale events both in terms of time and frequency, they turned to be undetected. Big events have the tendency to dominate small events, such that the small events go undetected [8–10]. The role of Topic Detection and Tracking for static documents has been discussed in the past, but for social network analysis there are some additional aspects to take into account such as real-time requirements, noise, fragmentation, and burstiness [5].

This paper undertakes to detect the influence of these aspects on event detection by observing the nature of the input data, its pre-processing, and examining the topic detectability of the selected algorithms. For this paper, tweets on the Oscars event are collected using some seed words, with the objective to detect the characteristic terms and subjects that explain the event. The selected data have some important characteristics that cover the domain of the film industry (the Oscars awards 2018). This dataset is selected for some important reasons to address when working on short texts. It contains significant events representing people or work-of-art who gathered much attention, and it also includes minor events representing those in the nominations but did not win awards and had less audience. Ground truths were produced using media reports, which gained more attention. It is desired to observe the performance of topic detection algorithms on this dataset.

The main contributions of this work can be summed up as follows:

- A comparison of unsupervised topic detection and tracking (TDT) methods to check their performance on more unlabeled heterogeneous dataset, the Oscars 2018, as many techniques work well on focused datasets but not on noisy datasets. For this purpose, 2,160,738 tweets related to the Oscars event are collected, which will be available publicly for further research.
- A study of the influence of various factors such as the type of input data and pre-processing on the quality of topic detection algorithms.

For conciseness, several abbreviations are introduced, which can be found in Table 1.

The rest of the article is carried out in the following manner.  Section 2 describes the literature review of the state-of-the art techniques used for event detection.  Section 3 presents the comparative analysis of event detection algorithms and the pre-processing step.  Section 4 illustrates the results and experiments and Section 5 concludes the paper.

## 2. Related Work

Event detection from the data stream is one of the active research fields and is the central theme of the Topic Detection and Tracking (TDT) domain. Data streams from social media, emails, blogs, online chats, and product reviews are collected and used for research purposes. Many approaches have been proposed for event detection tasks, focusing on text streams from social microblogs like Twitter. This section focuses on unsupervised techniques for event detection, such as probabilistic topic models, feature-pivot, and document-pivot.

A survey was conducted on Twitter-based event detection approaches and categorized as term-interestingness, topic modelling, and incremental clustering [4]. They concluded that incremental clustering techniques are more computationally effective than term-interestingness and topic modelling. Term-interestingness approaches work on the frequently co-occurring terms by calculating their tf-idf score. Some selection methods were employed to reduce the number of terms; every term is recognised by a named entity recognizer (NER) as a person, name, and location. The identification of interesting keywords impacts term selection methods, and it gives different results and often measures misleading term correlations. Topic-modelling approaches work on the assumption that there is always some hidden topic in the tweets, and it measures the probability distribution of each topic over the terms in the whole Twitter stream; in incremental clustering, some similarity metrics are used to measure the similarity between the cluster and the upcoming tweet. It is assigned to clusters by setting some threshold values. The method for the collection, grouping, ranking, and tracking of breaking news was proposed [11]. They collected 121,000 messages using Twitter API from public statuses and 33,000 messages from selected 250 users. They considered messages of only those users who used the headline news hash tag in their messages and considered two aspects for the detection of messages: (1) single message aspect and (2) timeline aspect. For the single message aspect, text-based information was considered and they extracted only those keywords that were nouns and verbs. For the timeline aspect, they considered bursty keywords and retweets. The proposed framework had two stages: story finding and story development. Story finding includes: (1) sampling—messages were fetched using some pre-defined queries to get real-time messages, (2) indexing—it was constructed based on the message content, and (3) grouping—similar messages were grouped together by comparing their tf-idf. They used the Stanford Named Entity Recognizer (NER) for grouping the proper nouns and they concluded that giving proper nouns more weight improves the similarity comparison of short texts. Real-world events or non-events are distinguishable from Twitter streams [12]. Real-world events include widely world occurrences, e.g., presidential inauguration, earthquakes, football matches, musical concerts, etc. On the contrary, non-event messages reflect videos, memes, opinions, personal thoughts, and information trending on Twitter but do not show any world occurrence. They used the online clustering algorithm whose threshold value was tuned in the training phase to form the clusters of the Twitter stream. Using certain features that include temporal, social, topical, and Twitter-centric, they identified various aspects of the clusters. They collected 2,600,000 Twitter messages and used human annotators for labeling the training and testing phases. They employed a variety of classifiers and the support vector machine yielded the best performance. There is a proposal for the detection of life events, which are a subset of events [3]. Marriage, graduation, birthdays, travel, job, and career change are a few examples of the life events that only affect an individual's life. They suggested that the frequency of life events is lower than other events, such that semantic feature consideration and temporal stacking are helpful in detecting these events. An analysis of the real-time surveillance system of traffic events of the Italian road network demonstrates the effectiveness of event detection [10]. They labeled the tweets as traffic-related or not traffic-related. SVM was used for this binary classification problem achieving 95.75% accuracy and for the multiclass classification problem 88.89%.

A comparison of LDA and deep belief nets (DBN) for 20 news groups' dataset is made [13]. The results showed that the DBN outperforms the LDA due to its deep architecture and highly nonlinear dimensionality reduction features. Semantic-based supervised classification of tweets based on lexical knowledge resources and WordNet domain for classification is possible [14]. Another study explored the detection of scientific tweets by analysing 2.63 million scientific tweets and investigated user account types and their geographical location using a feature-based approach [15].

Different probabilistic, pattern-based, machine learning-based, and clustering-based approaches have been proposed for event detection tasks. Existing approaches have some limitations for the event detection task in short texts. Pattern-based approaches have the drawback of scalability because it requires large event patterns which is cost prohibitive, whereas machine learning approaches first require feature engineering, i.e., extracting features from dataset as inputs to the classification models. Clustering approaches need some prior knowledge, e.g., number of clusters and similarity measures for finding similarity between clusters. Clustering approaches also have threshold settings and fragmentation issues. Second, traditional vector space models (VSM) were used for document representation. The drawback of VSM is that they do not distinguish the similar words of different events [16]. It is also observed that the temporal relationships between terms are no featured; hence, event detection methods lose an important feature. There have been models that seek to overcome these problems [17, 18]. In general, there have been issues of accuracy and efficiency in event detection [19].

## 3. Event Detection Approaches

### 3.1. Latent Dirichlet Allocation (LDA)

The topics underlying text corpora are extracted using probabilistic topic models. A topic model, in general, is a Bayesian model that correlates a probability distribution over topics with each document, which is a word distribution. LDA is a frequently applied probabilistic generative model; it is used in many machine learning applications. It is assumed that each document has a mixture of topics, and each topic is a mixture of words. LDA works by preserving the probabilistic relationship of words and topics while mapping the high-dimensional word space to the low-dimensional topic space [20]. In the view of LDA, each document is denoted by *d*_*m*_ and the number of words *N*_*m*_ in the corpus *D* is consisted of number of K different topics which constitutes the *K*-dimensional “document-topic” distribution *θ*_*m*_. Topics are formed by a mixture of vocabulary words *V* and constitutes *V*-dimensional “topic-word” distribution *φ*_*k*_[20].

As shown in Figure 1, LDA assumes the following generative process for a corpus D:

(1) Choose *θ*_*m*_ ~ *Di*  *r*(*α*) for the “document-topic” distribution on all *K* topics, where *α* is the parameter that defines the prior observation of the “document-topic” count.
(2) Choose *φ*_*k*_∼*Di*  *r*(*β*) for the “topic-word” distribution on all vocabulary words *V*, where *β* is the parameter that defines the prior observation of the “topic-words” count.
(3) Every word *w*_*i*_ in the document *d*_*m*_, 1 ≤ *i* ≤ *N*_*m*_, illustrate a topic *k* ~ *θ*_*m*_, and a word *t* ~ *φ*_*k*_[20].
(4) Collapsed Gibbs Sampling: LDA is trained to learn the topic-word distribution for each topic *k*, and it can be used to deduce the document-topic distribution for any new document. A collapsed Gibbs sampling (CGS), a Markov Chain Monte Carlo (MCMC) method, is an algorithm used to train the LDA. It is computationally effective and more precise than the standard Variational Bayesian Inference for LDA [5]. It works by generating samples of topics for all the words in the document *D* and then it performs the Bayesian estimation for topic-word distribution which is based on the sample topics. Initially, each word *w* is assigned randomly to topic *kϵK* and the information about the word-count *n*_*m*_^*k*^ and *n*_*k*_^*t*^ is computed which refers to the number of occurrences of topic *k* with the words of document *d*_*m*_ and the number of occurrences of words *t* with the topic *k*, respectively. In the next step, multinomial distribution P=[*p*_1,..,_*p*_*k*,…,_*pk*] is used to update the topic assignment for each word *wϵ*  *D*. Each part of P can be calculated by
  (1) $$\begin{array}{c} p_{k}\propto \frac{n_{k}^{t}+\beta }{\sum_{t=1}^{V}\left(n_{k}^{t}+\beta \right)}\times \frac{n_{m}^{k}+\alpha }{\sum_{k=1}^{K}\left(n_{k}^{t}+\alpha \right)}, \end{array}$$
where *p*_*k*_ defines the probability that topic *k* is sampled. After the given iterations, the process stops and it gives the topic samples *z*. The topic samples *z* and words *wϵ*  *D* are used to estimate the topic-word distribution *φ*_*k*_. Each part of *φ*_*k*_ can be calculated by
  (2) $$\begin{array}{c} \text{E}\left[\varphi_{k}^{t}|\text{z},\text{w}\right]=\frac{n_{k}^{t}+\beta }{\sum_{t=1}^{V}\left(n_{k}^{t}+\beta \right)}. \end{array}$$

### 3.2. Document-Pivot Topic Detection (Doc-p)

These techniques work by clustering the documents based on their textual similarity using similarity metrics such as Euclidean distance, Pearson's correlation, and cosine similarity. A threshold value is specified for measuring the similarity between document clusters. If the similarity between the document and the document in the collection is the same, both are added into the same cluster; otherwise, they are grouped in different clusters. Each generated cluster represents a topic. In this approach, tweets are represented as a bag of words representation using the tf-idf, which evaluates how important a word is to a document. It ignores the text's temporal, semantic, and syntactic features and suffers from dimensionality when the text is too long. The similarity between tweets is compared based on their tf-idf vector with the tf-idf vector of the first item and with the frequently occurring terms in each cluster. These incremental clustering approaches require suitable parameter settings. It will suffer from a mixed topic problem if the threshold value is too low, and a fragmentation problem will occur if the threshold value is too high. Fragmentation is the general problem in these methods: many clusters will represent a single topic. For short posts, the similarity of two items is usually one or close to one (1 or 0.8). Few researchers proposed the method for computing the similarity between documents by modifying the Local Sensitivity Hashing (LSH), which can efficiently provide the nearest neighbours concerning cosine similarity in an extensive collection of documents. The performance of document-pivot for tweets is not guaranteed because of the production of sparse vectors [8, 21].

### 3.3. Feature-Pivot Topic Detection (Feat-p)

Feature-pivot approaches were first developed for the analysis of timestamped document streams which treat an event as a bursty activity and emphasize specific terms. The concept behind these approaches is that when an event occurs, certain terms experience an abnormal increase in their frequency. These terms might be entities, nouns, verbs, or adjectives that burst throughout a certain period of time. As a result, most techniques in this area first find the bursty terms and then cluster them together for the extraction of events [5]. These methods require large documents because they rely on modelling the features in time [22]. The method proposed by [23] aimed at finding the bursty terms in a certain time window using the probability distribution of documents that contain those terms. After the bursty terms have been identified, they are clustered using a probabilistic co-occurrence model. In this case, LDA is used after the identification of bursty terms.

### 3.4. Soft Frequent Pattern Mining (SFPM)

Frequent pattern mining refers to a set of techniques that are able to find the co-occurring terms in big data. It plays an important role in finding the patterns from databases or transactional datasets. The first task of FPM is to find the frequent pattern itemsets that are calculated for each word and ignore the words with frequencies below a specific threshold. Sort the patterns based on their frequency and co-occurrences. After the extraction of frequent pattern itemsets, the next step is to create association rules and confidence rules (Association Rule Mining). The Apriori Algorithm is the most generally used technique for frequent pattern mining, but it has the disadvantage of requiring numerous scans of the database to count the support of the itemset, which is a time-consuming procedure and if the database is large, it would use a significant amount of disc I/O and CPU resources. Frequent pattern growth (FP-Growth) is the upgraded version of the Apriori Algorithm; it scans the database only twice and uses tree structures to store all the information. It creates a large number of itemsets directly from the tree and employs the divide and conquer technique to extract the frequent itemsets. It uses support and lift measures to rank the frequent patterns. Another upgraded version of FP-Growth is called soft frequent pattern mining (SFPM) that considers both the co-occurrence of two terms and the relationships between several terms. SFM begins with a single-term set S and then greedily grows it by computing the distance of each word to the set S. This operation is continued once the resemblance among the set S and the following term falls below a specific level [5, 24].

### 3.5. Singular Value Decomposition and *k*-Means Clustering (K-SVD)

SVD is a dimensionality reduction mathematical technique that works with matrices of data. The goal of SVD is to extract useful information from texts. The dimensionality reduction approach converts large matrices into smaller dimensions to compile a summary of the bulk of the data within that source matrix. In text mining, sparse term frequency matrices show mathematically the number of real-word frequencies in the documents. In techniques like LSA, SVD is employed in semantic analysis. In order to figure out the underlying meaning of terms in different documents, SVD decreases the dimensionality of the input matrix (total count of input documents divided by the total of terms to be evaluated) to a smaller space (a matrix of much shorter length of minimal data points), where each successive component reflects the most substantial amount of variability (means no fixed patterns vary a lot) between terms and documents. Now SVD works by computing an equation using 3 matrices that captures the information about data. In equation *X* = USV, the SVD of matrix *X* of size (*n* × *p*) (n is number of inputs and *p* is number of terms selected) will be calculated by computing equation USV, where S is the singular matrix of size (*n* × *p*). Consider singular values to be the most important values of the matrix's various features. *U* is the matrix of eigenvalues (eigenvalues show the directions of maximum spread or variance); it basically captures the information on rows of data. *V* is the matrix of eigenvalues that shows/captures the information on columns of data. With all these three matrices covering the rows, column information as well as the spread of variance, SVD tries to create a final relatively denser matrix than the initial one to show the association and meaning of terms across documents. SVD is the most widely used technique nowadays in NLP to analyse large terms across different documents [25–27].

*k*-means is the most extensively used unsupervised learning cluster-based algorithm in real-world pattern recognition applications [28, 29]. Because of its basic and easy-to-implement features, *k*-means is commonly employed in clustering. The objective behind *k*-means is to partition the dataset into *k* clusters that are pre-defined. The most important step is to define the centroid in each cluster, as different centroid positions in the dataset yield varied outcomes. Clusters with widely apart centroids are seen to be a preferable option for creating unique clusters. The distance from cluster *c* is used to allocate data points to clusters. The distance can be calculated using the Euclidean distance, Manhattan distance, Chebyshev distance, etc [30]. Within the clusters, the algorithm aims to decrease the squared distance [28]. After all of the data points have been assigned to clusters, the first iteration is finished, and the next step is to choose various *k* centroid centres until the centroid position does not change anymore. The approach is affected by the initialization phase and suffers from the problem of prior information of *k* clusters [31]. Although a lot of work has taken towards addressing these issues, it still needs to be improved.

## 4. Event Detection from Twitter Streams

In this section, after the problem statement is defined, the pre-processing steps are presented.

### 4.1. Problem Statement

Event detection in tweets for real-time data is undertaken. Tweets are made up of words, terms, or keywords and represent user-centred scenarios. Seed words are chosen to initiate the filtering process and narrow the analysis to only those posts that contain those seed words. The resulting outcome of the algorithms is a list of keywords that define the event detected in the Twitter stream. This setup necessitates gaining domain knowledge of the field of interest to select the initial seed words. Despite the fact that it requires preliminary human input, this framework is generic and may be applied to any topic or event.

### 4.2. Data Pre-processing

Users' posts are extremely chaotic in nature, containing formal and non-English terms, retweets, URLs, and symbols. It is necessary to pre-process the raw data collected using seed terms before beginning the event detection process. Pre-processing is a necessary process as it contributes in achieving high accuracy. The techniques used to pre-process the data are as follows:

- Case folding: Changing all the letters to lower case.
- Cleaning and Tokenization: Tokenization is the process of turning data into more valuable pieces of information. URLs, hashtags, mentions, retweets, emojis, and smileys are tokenized and removed.
- Stop words Removal: All the stop words are removed from the tweets making them more useful.
- Non-English Words: All the non-English words are removed.
- Removal of columns with length less than three.

Apart from these pre-processing steps, the dataset is selectively cleaned by removing some keywords based on subject knowledge. The removed keywords are listed in Table 2.

Figure 2 shows the word cloud after the pre-processing step. The words with high frequency are displayed in a larger font than words with a lower frequency.

## 5. Experimental Evaluation

In this section, the performance of the techniques on the Oscars 2018 dataset is tested and discussed. Section A provides a detailed overview about the used dataset, Section B describes the evaluation measures used to test the performance of the techniques, and section C provides the experimental results.

### 5.1. Dataset

The data for this study were gathered from the Twitter stream for one of the major events, the Oscars 2018, awards for artistic and technical merit in the film industry. The real-life event was held on 4th March 2018 GMT-8 at 5:00 pm. The dataset was collected a week before the event started, from Monday, February 26th to Tuesday, March 6th, 2018. The tweets related to this event were collected using the statistic of top-hashtags Oscar academy award in 2017. The dataset contains a total of 2,160,738 tweets which include only those tweets having one or more chosen seed words and keywords. Only English tweets are selected so that there are a total of 1,302,275 tweets in the dataset. The frequency graph of the whole dataset is given in Figure 3. From the graph, it is clear that the audience sent most tweets on 4th and 5th of March.

The Oscars 2018 Twitter activity is depicted in Figure 4. It is depicted from the graph that most tweets were sent the day before and the day of the event. Most tweets were sent between 10:00 pm (4 March 2018) and 05:00 am (5 March 2018). There is a surprise dip at 03:00 am (5 March 2018).

The ground truth about the event was extracted using the news headlines reported during the event [5, 24]. The ground truth includes 20 events related to the Oscars, such as who hosted the event, who wore the best dress, who won for the best picture award, best director, best actor, best documentary, best original score, etc. Only those events that gained much attention; some of the events are described in Table 3. The tf-idf representation of the tweets is used after removing the stop words and the pre-processing step. The dataset used in this paper is available publicly. Table 3 shows the examples of the event ground truths collected using media streams.

### 5.2. Evaluation Measures

Evaluation measures are important aspects of analysing the performance of any method. Mostly, all evaluation methods are influenced by the data's type [32]. This paper used *T*-Rec, *K*-Prec, and *K*-Rec due to their popularity in event detection [5, 22]. These evaluation measures help us find the fraction of relevant and irrelevant instances. Relevance is the foundation for both precision and recall [33]. Precision is a metric of quality, whereas recall is a metric of quantity. High precision indicates that the algorithm provides more relevant results than irrelevant ones, and high recall indicates that the method gives the majority of relevant results.

 
*Topic Recall (T-Rec)*: The proportion of ground truth topics successfully recognised by an approach. It can be calculated as the number of successfully retrieved topics divided by the number of topics should have returned.
 
*Keyword Precision (K-Prec)*: The proportion of the accurately extracted keywords out of the total number of keywords for the topics matched to some ground truth topic. It is calculated as the number of successfully retrieved results divided by the number of results returned.
 
*Keyword Recall (K-Rec)*: The proportion of the accurately recognised keywords over the total number of keywords of the ground truth topics. *K*-Rec is calculated same as *T*-Rec.

### 5.3. Experimental Results

*T*-Rec, *K*-Prec, and *K*-Rec are computed using ground truth annotations. First, they are computed on five numbers of topics. The dataset was pre-processed by eliminating the stop words, URLs, numbers, and non-English words. The Oscars dataset mainly consists of events about the celebrities' success, failure, performance, speech and their dressing sense, etc. The tf-idf was calculated for the pre-processed dataset and used as input features to these methods. The output of each method was a set of keywords that comes under the same cluster. The ground truth topics were 20 and results are computed up to 25 numbers of topics as the performance of all methods started to decline.  Figure 5 shows the graphical representation of the dataset obtained by K-SVD. It is observed that the resultant clusters increasingly overlapped with the number of clusters. The micro-averaging method is used to calculate the evaluation metrics.

The results of T-Rec, K-Prec, and K-Rec are given in Table 4. It is observed that when the chosen topics were 5 and 10, SFPM, Doc-p, and K-SVD produced better results. LDA and Feat-p did not perform well; both of the methods have low *T*-Rec, *K*-Rec, and *K*-Prec compared to other methods. SFPM yields the highest score among all the other methods. One reason for its high performance is that it captures the pattern in the dataset. K-SVD also performed well as it computes the similarity measures, which calculate the distance between the centroid and the other keywords. If the calculated distance is less to the centroid, it is assigned to the same cluster; otherwise, it forms another cluster. If the resulting event contains 80% of the keywords matched to some event in the ground truth event, it is considered successfully detected. SFPM yields the highest keyword precision and keyword recall than the other methods. It is because it searches for frequent patterns that come along together in the whole dataset. LDA and Feat-p have not performed well as the other methods. LDA can perform well on highly focused events, but it performs poorly when dealing with more noisy events, which are present in the Oscars dataset [5]. Due to LDA, Feat-p also yielded poor results, resulting in noisy event descriptions. The important observation here is that the pre-processing of input features also matters as selective removal of some keywords results in more appropriate event description. The removed keywords are those which occurred frequently and do not add meaning to event description but are noisier to use. Those keywords are captured from words cloud. It requires little effort but it's helpful in the identification of characteristic terms and subjects that describe the event.

Figures 6–8 show the *T*-Rec, *K*-Prec, and *K*-Rec of LDA, K-SVD, Doc-p, Feat-p, and SFPM.  Figure 6 shows that SFPM has the maximum *T*-Rec of 1, but when the number of topics grew to 25, it decreased to 0.7, implying that the strategy is successful. The lowest *T*-Rec of 0.5 is obtained by LDA and Feat-p.

All five approaches' *K*-Prec is shown in Figure 7. *K*-Prec was found to be maximum when the number of events was five, and it began to deteriorate as the number of topics increased. The highest *K*-Prec is 1 for SFPM, while the lowest is 0.5 for Feat-p, Doc-p, and LDA in this example. The lowest keyword precision in K-SVD is 0.7.

Figure 8 depicts *K*-Rec, and SFMP outperforms all other techniques, with a score of 1 in the best scenario and 0.6 in the worst. LDA and Feat-p have the lowest *K*-Rec of 0.4.

The experimental results show the better performance of *K*-Prec over *K*-Rec as there is a trade-off line between both metrics. One might assume that as the recall increases with model size, the precision decreases. However, this trade-off occurs in a small number of circumstances and does not result in a significant loss of precision. In most topic model types, increasing the number of topics leads to a minor loss in precision or even a small increase in precision [34]. In the Oscars 2018 dataset, precision and recall started to decline as the number of clusters increased; the explanation is that the formed clusters were referring to more and redundant events. Overall, the precision of all methods is high, indicating that the detected results are relevant, while their recall is low, indicating that most of the relevant results are not identified rather they are present in the ground truth topics.

Figures 9–12 illustrate some of the clusters obtained by the Doc-p method. Keywords are shown as features and the score shows the frequency of these keywords in the formed clusters.

All experiments are conducted with the default values of parameters of all methods. There are many parameters that can be tuned to obtain better results. Tf-Idf minimum and maximum values affect the resulting output. It's important to choose min tf-idf and max tf-idf carefully. In SFPM, a parameter min-support is used which can be adjusted manually. By varying the value of min-support, better clusters are formed. For the identification of the optimal number of clusters in the *k*-means algorithm, one can use the elbow method to see if it plots different clusters. Figures 13 and 14 show the elbow method created 10 and 15 clusters.

SVD and principal component analysis (PCA) both are used for dimensionality reduction. The shape of the dataset is visualized by forming different clusters. The tuning parameters of the LDA are number of topics, learning rate, and maximum iterations. All these hyperparameters are helpful to obtain better performance.

## 6. Conclusion

In this paper, a new and interesting dataset of real-life event, the Oscars 2018, is presented for text mining. It is collected from Twitter and used for research. The dataset allows a performance comparison of Topic Detection and Tracking (TDT) methods in terms of *T*-Rec, *K*-Prec, and *K*-Rec. The ground truth is mainly composed of 20 events that were gathered from news headlines. The 20 events are all related to the Oscars 2018. Events corresponding to the ground truth are investigated due to their importance as they emerged over time and the attention they sought. SFPM performed the best compared to LDA, Feat-p, Doc-p, and *K*-SVD in all three metrics. SFPM achieved the highest value of 1 on 5 topics for all three metrics. The lowest values were 0.7, 0.7, and 0.6 on 25 topics for *T*-Rec, *K*-Prec, and *K*-Rec, respectively. When the number of topics were increased to 25, all of the methods' performance started to deteriorate, forming duplicated and overlapped clusters. All methods obtained a better *K*-Prec implying that the most relevant results are produced. The low *K*-Rec implied most of the relevant topics remained undetected. All methods work well on the selected dataset and are generic in nature. This study has certain limitations in the sense that it investigates only the major events, i.e., those that gained much attention at the time of their occurrence. Minor events are not investigated. Also, the study does not cover all of the ground truth topics collected for the Oscars 2018 dataset. As a future work, strategies to increase the overall methods' performance will be investigated.

## Figures and Tables

**Figure 1:** LDA graph model.

**Figure 2:** Word cloud after pre-processing. It illustrates the nature of the dataset used.

**Figure 3:** Frequency graph of the Oscars 2018 dataset by dates. The real-life event was held on 4th March 2018.

**Figure 4:** Twitter activity of the Oscars 2018 event.

**Figure 5:** A graphical representation of the Oscars dataset using K-SVD for 5, 10, 15, and 20 clusters. When *k* = 5 and *k* = 10, the generated clusters are distanced from one another and distinct; however, when *k* = 15 and *k* = 20, the formed clusters are overlapped. (a) Clusters = 5. (b) Clusters = 10. (c) Clusters = 15. (d) Clusters = 20.

**Figure 6:** Topic recall of LDA, K-SVD, Doc-p, Feat-p, and SFPM.

**Figure 7:** *K*-prec of LDA, K-SVD, Doc-p, Feat-p, and SFPM.

**Figure 8:** *K*-rec of LDA, K-SVD, Doc-p, Feat-p, and SFPM.

**Figure 9:** Cluster 1 (best picture award Shape of water, as mentioned in Table 3) present in the ground truth topics. It demonstrates the effectiveness of the document-pivot strategy.

**Figure 10:** Cluster 2 (Meryl Streep dressed fairy godmother Shrek) present in the ground truth topics.

**Figure 11:** Cluster 3 (best animated feature film Coco) present in the ground truth topics.

**Figure 12:** Cluster 4 (Meryl Streep, Tiffany Haddish, Margot Robbie, and Jennifer Lawrence beautiful dressed) present in the ground truth topics.

**Figure 13:** *k*-means elbow method where *k* = 10. The elbow approach chooses an optimal value of *k* depending on the distance between data points and their associated clusters using the sum of squared distance (SSE). We picked a *k* value where the SSE started to flatten out and an inflection point appeared.

**Figure 14:** *k*-means elbow method where *k* = 15.

**Table 1:** Description of frequently used abbreviations.

Abbreviations	Description
Doc-p	Document-pivot
Feat-p	Feature-pivot
K-SVD	Singular value decomposition and *k*-means
LDA	Latent Dirichlet allocation
SFPM	Soft frequent pattern mining
*K*-Prec	Keyword precision
*K*-Rec	Keyword recall
*T*-Rec	Topic recall
Tf-idf	Term frequency-inverse document frequency

**Table 2:** List of keywords that were manually removed because they were not useful in generating meaningful clusters. Insightful observations can aid in the extraction of useful data.

People	Guarding	Red	Pay	Much
Black	Time	Carpet	Oh	Movies
Night	Things	Need	List	Well
Hey	Watch	Years	See	Still
Awards	Full	Tonight	Will	Let
Great	Man	Check	Live	Sign
Make	Yes	Double	Many	Room

**Table 3:** A list of ground truths collected from news headlines for the event, the Oscars 2018.

Story	Keywords
Shape of water won the best picture award	Shape, water, best, picture, award
Frances Macdormand won Oscar for best actress	Frances, Macdormand, won, oscar, best, actress
Guillermo Toro accepts best director for Shape of water	Guillermo, Toro, best, director, Shape, water
Michael Keegan gave happy reaction on Jordan Peele wins Oscar	Michael, Keegan, happy, reaction, Jordan, Peele
Meryl Streep dressed fairy godmother Shrek	Meryl, Streep, dress, fairy, godmother, Shrek
Gary Oldman best actor for darkest hour	Gary, Oldman, best, actor, darkest, hour
Coco won award for best animated feature film	Coco, won, best, animated, feature, film
Jimmy Kimmel talked on women harassment	Jimmy, Kimmel, talked, women, harrasment
Mcdormand speech powerful words “inclusion rider”	Mcdormand, speech, powerful, words, inclusion, rider
Dunkrik won three sound and editing Oscars	Dunkrik, won, three, sound, editing, Oscars
Kobe Bryant acceptance speech	Kobe, Bryant, accenptance, speech
Police investigates theft of $150000 Oscars dress won by Lupita Nyongo	Police, investigate, theft, Oscars, dress, won, Lupita, Nyongo

**Table 4:** Topic recall, keyword precision, and keyword recall of all the methods.

Methods	Number of topics	Topic recall	Keyword precision	Keyword recall
LDA	5	0.6	1	0.6
K-SVD	5	0.8	1	1
Doc-p	5	1	1	1
Feat-p	5	0.6	0.8	0.6
SFPM	5	1	1	1

LDA	10	0.8	0.7	0.7
K-SVD	10	0.8	0.8	0.8
Doc-p	10	0.8	1	0.8
Feat-p	10	0.7	0.7	0.6
SFPM	10	0.8	0.9	0.8

LDA	15	0.5	0.7	0.5
K-SVD	15	0.7	0.8	0.7
Doc-p	15	0.5	0.9	0.5
Feat-p	15	0.5	0.7	0.5
SFPM	15	0.8	0.9	0.8

LDA	20	0.6	0.6	0.5
K-SVD	20	0.7	0.8	0.6
Doc-p	20	0.6	0.8	0.5
Feat-p	20	0.6	0.6	0.5
SFPM	20	0.8	0.9	0.8

LDA	25	0.5	0.5	0.4
K-SVD	25	0.6	0.7	0.5
Doc-p	25	0.5	0.5	0.5
Feat-p	25	0.5	0.5	0.4
SFPM	25	0.7	0.7	0.6

## Data Availability

All data generated or analyzed during this study are included in this published article.
